# Clinical Application of Peritoneal Dialysis Catheterization without Capsular Puncture Technique

**DOI:** 10.1155/2022/2733659

**Published:** 2022-09-19

**Authors:** Zhifeng Wei, Xiaoli Han, Yunxia Zhi, Junfen Liu, Xing Pan, Shengjun Liu

**Affiliations:** The First Affiliated Hospital of Hebei North University Nephrology Department, Zhangjiakou, Hebei 075000, China

## Abstract

**Objective:**

To summarize the advantages of peritoneal dialysis (PD) catheters without capsular puncture (only one pneumoperitoneum needle) puncture technique conducted by our center.

**Methods:**

The study examines the clinical data of PD patients (including the general situation of patients, intraoperative and postoperative characteristics, and complications) undergoing pneumoperitoneum needle catheterization from January 2019 to May 2021 in the Department of Nephrology at the First Affiliated Hospital of Hebei North University (the largest peritoneal dialysis center in Zhangjiakou).

**Results:**

A total of 153 surgical cases were collected. There were 91 males and 62 females. The mean (± standard deviation) age was 56.1 ± 18.6 years, and the mean (± standard deviation) follow-up time was 16.7 ± 8.2 months. The average operation time was 30.33 minutes with a standard deviation of 14.80 minutes. The length of abdominal incision is 2.38 ± 0.42 cm, and the blood loss was about 26.3 ± 9.2 ml, including 2 cases of laparoscopic reposition of drift tube, 0 case of pipe blockage, 3 cases of fluid leakage, 1 case of peritoneal dialysis catheter tunnel infection, 4 cases of outlet infection, 12 occurrences of peritonitis, 121.3 patient months in peritonitis, and 0 times in omentum wrapping without bladder injury, incisional hernia, or intestinal injury.

**Conclusion:**

Relative to open operation, the peritoneal dialysis (PD) catheters with pneumoperitoneum needle puncture technique has the following advantages: simpler operation, shorter operation time, less bleeding, less injury, less complications, and higher safety. Moreover, there are no additional costs compared with open operation. Thus, the technique is recommended for clinical applications.

## 1. Introduction

Peritoneal Dialysis (PD) is one of the most important techniques of renal replacement therapy for end-stage renal disease (ESRD) patients [1]. ESRD, which refers to the end stage of various chronic kidney diseases, is similar to uremia in concept, but the diagnostic criteria are different. It is generally believed that the diagnosis can be made when the pellet filtration rate drops below 15 ml/(min.1.73m^2^). More than 270,000 ESRD patients worldwide have been treated with peritoneal dialysis so far [2]. And the annual growth rate of PD (8%) [3] has exceeded the growth rate of hemodialysis patients (6%-7%) [4]. PD catheters is the “Lifeline” for PD therapy, so its patency and safety are essential [5]. Therefore, successful peritoneal dialysis catheterization is necessary for successful peritoneal dialysis [6]. A large number of experts at home and abroad have made continuous innovations in the methods of PD Catheterization, aiming for less trauma to patients, longer service life of catheters, less complications for patients, and lower cost of treatment. The technique has evolved from the initial open catheterization and laparoscopic catheterization to the more recent Seldinger technique and trocar technique [7].

There are three types of renal replacement therapy for patients with ESRD, including hemodialysis, peritoneal dialysis, and kidney transplantation. Peritoneal dialysis is safe and effective, simple to operate, does not need to rely on machines, and is not easy to cross infection. Biocompatibility is not easy to appear allergic reaction, small impact on the cardiovascular system, and other advantages. When kidney transplantation is not the first choice for ESRD patients, peritoneal dialysis can be prioritized, especially for patients with heart failure and chronic cardiorenal syndrome, excluding contraindications related to peritoneal dialysis. The key to the successful development of peritoneal dialysis is the establishment of access. At present, there are three methods commonly used to establish access, which are surgical incision, percutaneous puncture, and laparoscopic method. Different catheterization methods have their own advantages and disadvantages.

Most patients with ESRD have abnormal cardiac function, and surgical incision catheterization takes a long time. At the same time, pain stimulation during muscle layer separation and purse-string suture can induce heart failure symptoms such as chest tightness, asthma, and gastrointestinal symptoms such as nausea and vomiting. However, the catheterization time of peritoneal dialysis is short, there is no need to separate the muscle layer and involve the peritoneum, the pain and stimulation are small, the patient's tolerance is increased, and the cardiac function is less affected. At the same time, surgical incision catheterization cannot be used as early as possible for peritoneal dialysis treatment, which prolonging the length of hospital stay. In addition, nephrology physicians in primary hospitals do not have the qualification of surgical catheterization and the lack of catheterization technology, which limits the development of peritoneal dialysis.

The advantages of peritoneal dialysis catheterization are as follows: no surgical assistance is required; shorten the catheterization time and reduce the surgical wound; relieve pain of patients; abdominal incision and purse-string suture are not required, and the probability of fluid leakage is reduced. The catheter technique has a high survival rate, and peritoneal dialysis can be started immediately. Low complication rate: the hospital stay is shorter and more economical.

In recent years, our center has made several improvements on the PD catheterization surgery, where we have achieved better clinical results by using the pneumoperitoneum needle catheterization. This paper details the techniques we have learned.

## 2. Data and Methods

### 2.1. Clinical Data

From January 2019 to May 2021, 153 patients with end-stage renal disease who received uncapsulated (only one pneumoperitoneum needle) peritoneal dialysis catheterization in the Department of Nephrology at Hebei North University were selected for the study. All patients included had clear indications for renal replacement therapy, no PD contraindication, and the operation was performed by the same surgeon, and the Tenckhoff straight tube was used. This study was approved by the hospital ethics committee, and all patients were informed and signed informed consent.

### 2.2. Method of Operation

#### 2.2.1. Preoperative Preparation

Patients were given routine skin preparation, enema, bladder emptying, and antibiotics to prevent infection. The pneumoperitoneum needle is shown in Figure 1.

#### 2.2.2. The Surgical Procedures

The patient was placed in the supine position, and a body surface marking line was drawn at the rectus abdominis muscle 10-12 cm above the pubic symphysis. The skin of the operation field was routinely disinfected, and 1% lidocaine was used for local infiltration anesthesia. The skin incision was about 2 cm, and the subcutaneous tissue was bluntly separated, the anterior sheath of rectus abdominis muscle was cut open, and the rectus abdominis muscle was bluntly separated, and the sheath of rectus abdominis muscle was exposed, as shown in Figure 2. The pneumoperitoneum needle needs to pass vertically through the rectus sheath and peritoneum. After pulling out the pneumoperitoneum needle, the hemostatic forceps slightly dilate the puncture opening to be close to the outside diameter of the peritoneal dialysis catheter. A guide wire was used to guide the peritoneal dialysis catheter to the rectus abdominis bladder (uterus) depression, then the guide wire was removed, and the anterior rectus abdominis sheath was sutured. A tunnel needle was used to establish a subcutaneous tunnel, the peritoneal dialysis catheter was withdrawn, and the subcutaneous tissue and skin were sutured. Finally, the incision and outer opening are covered with dressings, and a pressure bandage is worn on the abdomen. The surgical procedure is shown in the following figure.

The supine position described above refers to lying on the pillow with the head tilted to one side. Arms at the side of the body, legs naturally straight, and the pillow straight over the head of the bed. Rectus abdominis muscle was located on either side of the midline of the anterior abdominal wall. The rectus abdominis muscle is in the rectus abdominis sheath. It is a band shaped multiabdominal muscle, which is wide above and narrow below, and rises from the pubic symphysis and the pubic crest.

### 2.3. Observation Index

① Basic data of patients before operation (including age, sex, body mass index, hemoglobin, albumin, estimated glomerular filtration rate, history of abdominal surgery, and primary kidney disease); ② perioperative condition: operation time, incision length, intraoperative blood loss, time to start peritoneal dialysis, conversion to laparotomy, hospital stay after operation; ③ visual analogue scale score (VSA) was used to evaluate the pain degree of d0, D1, D2, and D3 after catheterization. ④ Intraoperative and postoperative complications: including PD drift tube, tube blockage, fluid leakage, exit infection, tunnel infection, peritonitis, and organ injury. ⑤ Survival rate of PD catheter technology: the PD tube removal due to complications, inadequate dialysis, peritoneal ultrafiltration, and other reasons from successful PD catheterization to the end of follow-up was observed, and the survival rate of PD catheter technology was calculated.

### 2.4. Dialysis Methods and Dose

According to their own conditions, patients chose automatic peritoneal dialysis (APD), daytime ambulated peritoneal dialysis (DAAPD), and continuous ambulated peritoneal dialysis (CAPD), and glucose peritoneal dialysis fluid produced by Baxter was used for PD fluid.

### 2.5. Statistical Methods

SPSS 21.0 software was used for data statistics, in which the measurement and count data were expressed in the form of (±s) and rate (*N*/%). The PD catheter survival curve was drawn by Graphpad Pism 5.0.

## 3. Results

### 3.1. Basic Data of Patients

A total of 153 surgical patients were collected in this study, including 91 males and 62 females, with an average age of 56.1 ± 18.6 years, including 57 patients with a history of abdominal surgery. The primary renal diseases were chronic glomerulonephritis in 84 patients (54.9%), diabetic nephropathy in 47 patients (30.7%), hypertensive nephropathy in 6 patients (3.9%), polycystic kidney disease in 3 patients (1.9%), and other renal diseases in 13 patients (8.5%). The basic data of the patients are shown in Table 1.

### 3.2. Perioperative Situation

All 153 patients with catheterization completed surgery successfully, and no patient was transferred to laparotomy. Specific details are shown in Table 2.

### 3.3. Pain Degree of Patients after Catheterization

The patient presented with moderate pain on the day after surgery and basically felt no pain 3 days after surgery. The score is shown in Table 3.

### 3.4. Intraoperative and Postoperative Complications

2 cases of laparoscopic reduction with drift tube occurred after surgery; 3 cases of fluid leakage; peritoneal dialysis catheter tunnel infection: 1 case; 4 cases were infected by export; peritonitis occurred in 12 patients (121.3 patient months). There were no bladder injury, incisional hernia, and intestinal canal injury in all cases (see Table 4).

### 3.5. Survival Rate of Catheter Technique

The follow-up time was up to January 2022; the longest follow-up time was 36 months, with an average follow-up time of 16.7 ± 8.2 months. There were 153 patients with catheter technique failure 3 times; 2 cases were catheter displacement, within 1 week after surgery. One case was peritonitis, which occurred 1 year and 3 months after surgery. The technical survival curve of the catheter is shown in Figure 3.

## 4. Discussion

PD is an important alternative therapy for patients with end-stage kidney failure. Due to its advantages such as simple operation, early retention of residual renal function, hemodynamics stability, and low risk of blood disease transmission, [8], the procedure has become the preferred alternative treatment for ESRD patients. The premise and guarantee for the smooth progress of PD must be the presence and smoothness of PD tube [9]. Common complications of PD catheterization include poor catheter position, drift tube, greater omentum encapsulation or blockage, poor drainage of dialysate, dialysate leakage, peritonitis, exit/tunnel infection, visceral injury, and hernia. These complications will not only increase the patient's pain and treatment costs; these patients will be not be suitable for PD. The incidence of noninfectious complications was closely related to the surgical procedures. The incidence of catheter drift in PD patients was reported to be 7.6%-16% [10, 11], and the incidence of greater omentum wrapping was 3.2%-27% [12–14]. In order to reduce the high incidence of postoperative complications, the researchers at home and abroad have been searching for the optimal catheterization for many years.

At present, there are three kinds of catheterization commonly used in clinic: open surgical catheterization, laparoscopic catheterization, and percutaneous catheterization. The percutaneous catheterization mainly includes Seldinger technique or Trocar technique. Different types of surgery also have their own advantages and disadvantages. Open surgical catheterization is the standard catheterization method commonly used in clinic [15]. Compared with surgical catheterization, laparoscopic catheterization is less invasive and more effective [16], but both of them require more surgical equipment and personnel, and they have high requirements on the patient's surgical tolerance. Trocar puncture and catheterization cost is relatively low, but the trauma is large, the safety of puncture is low, and the practicality is poor, which limits its clinical use. Seldinger puncture catheter method can be in bed, relatively simple [17] operation, especially suitable for emergency use [18], and minor damage, but the piercing suite expensive, blind wear easily puncture injury intestines, fat before the peritoneal cavity or failure cause [19, 20], clinical need ultrasound guided puncture [21], grassroots hospitals are not easy to promote. Seldinger catheterization does not require the cooperation of surgeons. The catheter is similar to the semilong-term hemodialysis catheter assembly, which is easy to operate, has short catheterization time and less trauma, and can be used for early peritoneal dialysis treatment and shorten the length of hospital stay. Nephrologists can be qualified through training. Many studies have shown that compared with Trocar, the operation time of Seldinger method is significantly shorter than that of surgical incision method. The shortening of operation time is mainly because there is no need to cut the anterior sheath of rectus abdominis muscle, no need to separate the muscle layer, no need to purse-string suture, etc. At the same time, because there is no need to open the abdominal cavity, all the incisions are smaller, the injury is reduced, and the patient's tolerance is enhanced.

Peritoneal dialysis catheters were placed in our center by PD catheterization without encapsulation (only one pneumoperitoneum needle). Because of the unique structure of the pneumoperitoneum needle, it can penetrate the abdominal cavity smoothly; the puncture feeling is easily sensed and will not damage the intestinal tract. And the pneumoperitoneum needle can be inserted vertically into the postsheath; because of the small opening of the peritoneum and the posterior sheath, no purse-string suture is needed, which can reduce the difficulty of the operation, shorten the operation time, and reduce the amount of bleeding during the operation, causing less pain to the patient. In addition, pneumoperitoneum needle can be fixed firmly in the peritoneal cavity of peritoneal dialysis catheter. The rate of leakage was only1.96%, no greater omentum encapsulation and organ injury, and the rate of peritonitis was 121.3 patient months, which was also lower than that reported in the literature. In addition, from the perspective of health economics, pneumoperitoneum puncture can reduce complications without increasing patient costs, which is especially suitable for primary doctors.

In conclusion, pneumoperitoneum needle puncture PD catheterization has the advantages of simple surgical process, short time, less bleeding, less patient injury, high safety, low rate of drifting tube and greater omentum wrapping rate, low infection rate of exit and tunnel, and economic benefits. Meanwhile, PD catheterization is widely applicable to a wide range of people and can be safely applied to emergency and elective peritoneal dialysis patients, which is worthy of clinical promotion.

## Figures and Tables

**Figure 1:** Gas meter puncture and multimode through-fold catheterization.

**Figure 2:** The procedure.

**Figure 3:** The technical survival curve of the catheter.

**(a):** 

Age (years old)	Sex (*n*)		BMI (kg/m^2^)	Hemoglobin (g/l)	Total serum protein(g)	Glomerular filtration rate (ml/min/1.73 m^2^)	History of abdominal surgery
	Male	Female					
56.1 ± 18.6	91	62	22.3 ± 6.85	89.4 ± 21.4	68	5.8 ± 2.5	57

**Table:** (b) Primary nephropathy *n* (%)

Chronic glomerulus nephritis	Diabetes kidney disease	Hypertension kidney disease	Polycystic kidney	Other
84 (54.9%)	47 (30.7%)	6 (3.9%)	3 (1.9%)	13 (8.5%)

**Table 2:** Perioperative conditions.

The length of the incision (cm)	The operation time (min)	Intraoperative blood loss (ml)	Transfer laparotomy [*n* (%)]	Start time of dialysis (h)	Hospitalization days (d)
2.38 ± 0.42	30.33 ± 14.80	26.3 ± 9.2	0	19.48 ± 5.37	12.36 ± 4.62

**Table 3:** VSA pain scores of patients ($\bar{x}\pm s$, min).

d0	d1	d2	d3
4.24 ± 1.35	2.31 ± 0.84	1.32 ± 0.46	0.21 ± 0.07

**Table 4:** Complications (*n*/%).

Drift tube	Blocking pipe	Leakage	The tunnel infection	Exit infection	Peritonitis	Viscera damage	The total incidence
2 (1.30%)	0	3 (1.96%)	1 (0.65%)	4 (2.61%)	12 (7.84%)	0	14.4%

## Data Availability

The dataset used in this paper are available from the corresponding author upon request.
